This article has been retracted.

# Evaluation of Cholesterol Thickness of Blood Vessels Using Photoacoustic Technology

**DOI:** 10.1155/2023/2721427

**Published:** 2023-04-12

**Authors:** Alaa Kassar Salih, Ala Hadi ALWAN, Maria Jade Catalan Opulencia, Herlina Uinarni, Firuza M. Khamidova, Mohammed Shakir Atiyah, Sura A. Awadh, Ali Thaeer Hammid, Zeinab Arzehgar

**Affiliations:** ^1^Al-Nahrain University, Baghdad, Iraq; ^2^Ibn Al-Bitar Specialized Center for Cardiac Surgery, Baghdad, Iraq; ^3^Ajman University, Ajman, UAE; ^4^Atma Jaya Catholic University of Indonesia, Jakarta, Indonesia; ^5^Pantai Indah Kapuk Hospital, North Jakarta, Indonesia; ^6^Department of Ophthalmology, Samarkand State Medical Institute, Samarkand, Uzbekistan; ^7^Tashkent State Dental Institute, Tashkent, Uzbekistan; ^8^Al-Manara College for Medical Sciences, Maysan, Iraq; ^9^Al-mustaqbal University, Babylon, Iraq; ^10^Imam Ja'afar Al-Sadiq University, Baghdad, Iraq; ^11^Department of Chemistry, Payame Noor University, Tehran, Iran

## Abstract

One of the primary indicators of plaque vulnerability is the lipid composition of atherosclerotic plaques. Therefore, the medical industry requires a method to evaluate necrotic nuclei in atherosclerosis imaging with sensitivity. In this regard, photoacoustic imaging is a plaque detection method that provides chemical information on lipids and cholesterol thickness in the arterial walls of the patient. This aspect aims to increase the low-frequency axial resolution by developing a new photoacoustic-based system. A photoacoustic system has been developed to detect the cholesterol thickness of the blood vessels to observe the progression of plaque in the heart's blood vessels. The application of the coherent photoacoustic discontinuous correlation tomography technique, which is based on a novel signal processing, significantly increased the cholesterol oleate's sensitivity to plaque necrosis. By enhancing the quality of thickness detection, the system for measuring the thickness of cholesterol in blood vessels has been reduced to approximately 23 microns. The results show that the phase spectrum peaked at 100 Hz at 58.66 degrees, and at 400 Hz, the phase spectrum was 46.37 degrees. The minimum amplitude is 1.95 at 100 Hz and 17.67 at 400 Hz. In conclusion, it can be stated that photoacoustic imaging as a method based on new technologies is of great importance in medical research, which is based on the use of nonionizing radiation to perform diagnostic processes and measure different types of body tissues.

## 1. Introduction

In recent years, imaging of different parts of the body has been able to play a significant role in the diagnosis of various diseases; consequently, many medical studies are being conducted in this field around the world. Various techniques, such as X-ray imaging or ultrasound and optical waves, or nuclear medicine imaging, have been developed to pinpoint the location of tumors, inflammation, or pain in various body tissues. Even if these techniques are proven to be effective, the most important factor in using them is the restriction on their use to patients. As a result of their high penetrating power, X-rays are utilized to radiograph organs. Since X-rays are classified as ionizing radiation, they are harmful to live tissues. Suppose a patient is exposed to high doses of radiation, even for a short time, the risk of radiation sickness increases, increasing the risk of cancer. However, in most medical applications, X-ray dangers are typically overlooked due to the images they produce. The image quality is poor in medical ultrasound imaging, which is nonionizing compared to X-rays. In addition, optical imaging methods are of poor quality due to the excessive scattering and attenuation of photons in living tissue. Therefore, utilizing a combination of imaging systems in the form of an integrated system and producing high-quality images is one of the modern techniques used to overcome the drawbacks of conventional medical imaging. Nonionizing radiation is electromagnetic and fields with photon energies below 10 eV, corresponding to frequencies below 3 PHz (3 × 1015 Hz) and wavelengths longer than 100 nm. The primary objective of both ionizing and nonionizing radiation protection is to safeguard human health and the planet from damage. For people, the priority is to protect all lives, but for the ecology, the objective is to safeguard species, ecosystems, and biota against harmful consequences. Also, when complete information about dangers associated with radiation absorption is lacking, safe handling means creating educated judgments. ICNIRP acknowledges that a comprehensive approach to safety against the harmful impacts of nonionizing radiation must include socioeconomic analyses [1].

Photoacoustic imaging, which combines optical systems with ultrasound waves, is one of these techniques. Noninvasive photoacoustic imaging in catheter systems and photoacoustic endoscopy is used to examine living tissues in the body without the problems associated with other techniques. Photoacoustic describes a physical phenomenon in which light wave energy is absorbed by a substance to produce sound waves. Fully optical imaging techniques, such as optical coherence tomography, provide high-contrast spectroscopy based on imaging targets' optical properties, particularly scattering coefficient [2]. However, their imaging depth is limited because not enough photons can be detected upon returning from subsurface targets. On the other hand, the spatial resolution of ultrasound imaging allows for depth penetration, but its contrast is limited because it detects targets based on device characteristics such as density [3]. By combining these two techniques, the contrast of photoacoustic imaging, which is based on the difference in optic absorption between targets and surrounding tissue, encrypts and transmits the generated information as acoustic signals. Photoacoustic imaging is a novel technique that combines the high contrast of optical imaging with the deep subsurface penetration and high spatial resolution of acoustic imaging [4]. Photoacoustic imaging produces a photoacoustic signal by absorbing infrared light near the first and second vibrational energy levels. The signal generated contains information that can be detected at a tissue depth [5]. Unlike optical tomography, the integration of near-infrared spectroscopy with ultrasound detection eliminates wave scattering issues [6]. By simultaneously utilizing the capabilities of the integrated systems, hybrid imaging techniques make it possible to improve the quality of the resulting images compared to what each system alone can produce. As a hybrid of ultrasonic imaging and optical imaging techniques, photoacoustic imaging, which uses the ultrasonic wave produced by the tissue after receiving a laser pulse to create medical images, has entered the field of medical research.

The photoacoustic imaging method provides images with optimal contrast and resolution for physiological and anatomical studies. This method can noninvasively image cells and arteries, detect normal tissue from cancerous tissue, and image the entire body in humans and animals because it does not utilize ionizing radiation. Owing to their close relationship with the physiological state of the tissue [7], the optical properties of biological tissue are generally important diagnostic parameters. Thus, photoacoustic imaging can compare the available information of its biological targets with the anatomical information provided by other common imaging techniques, such as X-ray imaging [8]. Photoacoustic imaging typically concentrates on the near-infrared spectrum between 700 and 1300 nm. This spectral region is popularly known as the optical window [9]. Electromagnetic waves can penetrate living organisms to the maximum depth possible. This is why photoacoustic techniques can be used in various fields, including biology, medicine, and the industrial sector. Photoacoustic techniques can be used in various fields, including biology, medicine, and the industrial sector [10]. The spatial resolution of a photoacoustic system is, by definition, the basis for determining the minimum lateral and axial lengths for bandwidth and optical wavelength [11]. Lateral resolution is the minimum detectable distance between two adjacent locations, which varies according to the size of the laser beam point. In this region, tissue chromophores and water have relatively low absorption coefficients but high effective scattering coefficients [12]. In addition, numerous tissue chromophores, such as hemoglobin and fat, have a unique absorption spectrum in this region [13]. Compared to an optical window, the absorption rate of water in the spectral region is less than 700 nm. Nonetheless, because the optical dispersion of water in this region is high, optimal adsorption on the substrate's target chromophores is less frequent. On the other hand, the optical dispersion of water decreases in the wavelength range above the 1,300 nm optical window. However, since water absorption is predominant, the target chromophores exposed to light transfer are less accessible [14].

Photoacoustic imaging techniques have been applied to imaging cancer, wound healing, brain disorders, and gene expression. Photoacoustic imaging has several good points, such as using nonionizing electromagnetic waves, having good resolution and contrast, using portable equipment, and partially measuring the signal. Optical and rf waves are used in photoacoustic imaging instead of electromagnetic waves at other wavelengths due to their advantageous physical features, such as deeper tissue penetration and enhanced contrast agent absorption. The combination of high ultrasonic resolution and outstanding picture contrast due to differential optical/rf absorption is extremely useful for imaging applications. In contrast to fluorescence imaging, where tissue scattering restricts spatial resolution with increasing depth, photoacoustic imaging has a better spatial resolution and greater imaging depth due to the less dispersion of the ultrasonic signal in tissue. In comparison to ultrasonic imaging, where the mechanical characteristics of biological tissues restrict tissue contrast, photoacoustic imaging provides superior tissue contrast, dependent on various tissues' optical properties. In addition, photoacoustic imaging is safer than other imaging methods, such as computed tomography and radionuclide-based imaging techniques, due to the lack of ionizing radiation. While the disadvantage is that focusing is limited to a specified depth [15].

In soft tissue optical imaging methods, optical images have a high contrast due to the electromagnetic wave's absorption interaction with the material. However, the spatial resolution is significantly reduced by using short wavelengths. In contrast, the ultrasonic imaging method, where the contrast of images is generally low due to low-speed changes, produces images with a very high resolution and greater detail from the study area during short ultrasonic wavelengths. Taking advantage of both optical and ultrasound imaging, the photoacoustic imaging method [16] aims to provide higher contrast images (compared to ultrasonic imaging) as well as better resolution and penetration depth (compared to optical imaging). Typically, the photographic, acoustic resolution of a tomograph is determined by the transducer's properties that receive the ultrasound. When a converter with a central frequency and a larger bandwidth is utilized, the highest resolution is achieved. Due to the high attenuation of ultrasound at high frequencies, ultrasonic transducers with a central frequency between 1 and 20 MHz are used for photoacoustic tomographic imaging of deep tissues. Photoacoustic waves are typically detected using piezoelectric detectors, which have high sensitivity and the ability to produce desired shapes and can be used for parallel detection. Recent efforts have been made to produce and employ ultrasonic-optical detectors, which may be more appropriate in this field due to their uniform amplitude response over a broad frequency range and optical transparency [17].

The average free path of photons in biological tissue is 1 mm, even in the near-red region. Because purely optical imaging techniques rely on multiple scattered light events before collecting information generated by a tracker, accurate depth-of-field imaging is difficult [18]. In photoacoustic imaging, it is anticipated that the total distance traveled by photons or the number of light scatterings required will be significantly lower than in fully optical methods [19]. The generated visual information is then decoded in sound pressure waves by the photoacoustic effect [20], whose propagation speed depends on the sound's distance from the detector. Because sound scattering is significantly smaller than optical scattering by two to three times the path length, photoacoustic signals can be easily detected from great distances [21]. High-frequency components of propagation signals carry minute information, while low-frequency components carry extensive data. The high-frequency components are easily compromised when signals must travel over great distances. On the other hand, low-frequency components can travel significantly greater distances without significant content degradation [22, 23].

A prompt treatment action requires early detection. Moreover, it needs reliable diagnostic tools capable of identifying disease development in its early stages and assessing the success of therapy in clinical settings. Photoacoustic imaging is a revolutionary technique that may diagnose diseases in their earliest stages and continually track their course. Methods for earlier detection and accurate evaluation of illness development are essential for improving clinical health results, prompt treatment, and effective changes to medications [24]. The axial resolution of photoacoustic pulses is dependent on the bandwidth of the applied ultrasonic transducer and the width of the laser pulse [25]. Combining a high-frequency converter with a low-frequency converter increases the axial resolution but destroys the photoacoustic signals in the imaging depth [26, 27]. Sufficient photon energy must reach the subsurface target absorber for high-resolution imaging, and ultrasonic signal attenuation must not severely limit imaging depth [28]. Several techniques [29, 30] have been developed to improve the axial resolution of photoacoustic systems. The two primary strategies in each case are the use of broadband converters with short excitation pulses and ultraprecise imaging methods [31]. In both instances, the axial resolution improves, penetrating more deeply due to its connection to high-frequency converters. Increasing modulation frequency increases axial resolution [32, 33].

Today, one of the fundamental requirements of medical science for diagnosing cardiovascular disease is utilizing a highly sensitive method for diagnosing atherosclerosis. Consequently, the necessity of the present study is elucidated. Utilizing a combination of imaging systems in the form of an integrated system and producing high-quality images is one of the modern techniques used to overcome the limitations of conventional medical imaging. Among these techniques is photoacoustic imaging. This study aimed to evaluate the efficacy of a photoacoustic-based system for detecting cholesterol thickness in the heart's blood vessels. In this study, the system for measuring the thickness of cholesterol in blood vessels was reduced to approximately 23 microns by improving the quality of thickness detection. Notably, the technique of coherent photoacoustic discontinuous correlation tomography, which is based on new signal processing, has been used to examine the sensitivity of oleate cholesterol in this regard.

## 2. Materials and Methods

Photoacoustic imaging combines optical and ultrasonic waves (the range of infrared waves). This method has the depth of penetration and appropriate contrast of ultrasound waves and the high resolution of light waves. Typically, photoacoustic imaging is performed in two ways [34]. Only photons are transmitted to the tissue of interest in the first method. After colliding with tissue, several photons are reflected, which can be collected with an optical lens. Other photons are absorbed by the tissue, resulting in tissue heating. Due to thermoelastic expansion and the resulting expansion, ultrasonic waves will be generated, which can be received by placing an ultrasonic transducer and reconstructing an image [35, 36]. In addition, the tissue's temperature rises due to the absorption of photons and their energy, proportional to the difference between the energy of the absorbed photons and the energy of the ultrasonic waves produced, which can be used for thermoacoustic imaging.  Figure 1 depicts how photoacoustic waves are generated. By sending a laser pulse and striking the tissue, as can be seen, some of the laser pulses are reflected, and others are absorbed by the tissue, causing thermoelastic expansion in the tissue and the propagation of ultrasound waves [37].

A device depicted in Figure 2 is utilized to demonstrate the highest achievable axial resolution. Using the shear algorithm, two integrated photoacoustic signals can be detected from flat absorption surfaces with different time delays. A Plexiglas wedge coated with a thin layer of cholesterol oleate was prepared to test the technique. The coating method is based on the melting of cholesterol oleate with indirect heat and forming a primary coating nucleus for the Plexiglas surface. Plexiglas (PG) was chosen as a substrate due to its low sound speed and greater impedance compatibility with the systems connected to it to reduce sound reflections at the boundaries. The laser excitation utilized an infrared light source with 1100 nm and a thermoelectric cooling system. Fiber optics and a collimator lens direct the laser's output beam to the sample chamber [38, 39]. The 10-megahertz-to-30-megahertz frequency range of the Python-generated waveform was loaded. A photoacoustic preamplifier receives a sinusoidal photoacoustic signal and then transmits it to the host computer. A cholesterol-coated wedge was submerged in a water tank with a wedge surface to simulate two photoacoustic signals with spatial and spatial correlations. Thus, the laser beam modulated to generate ultrasonic waves reaches the cholesterol-coated wedge surfaces. Using a micrometer, the wedge attached to the micrometer, which is all on the optical table, was moved at regular intervals. The point of contact of the laser radiation with the adjacent points was 46 micrometers in the direction of the laser radiation. Preparation of semitransparent PG specimens for laser irradiation reduced the generation of unwanted photoacoustic signals. The transmitted beam was stopped after passing through two layers of cholesterol oleate outside the vessel. By connecting the tip of the optical fiber to the radiation conduction and scanning system in position, signals from the sample to the transducer are transmitted simultaneously and proportionally. The algorithm will include the possibility of manual scanning by guiding the catheter tip with an external control system or automatic point-by-point collection and processing in the computer. Figure 2 depicts the methodology employed in this study.

The sample was examined using an Nd: YAG laser with a 1064 nm pulse to compare the present method to the pulse method. In the same configuration as the present method, Nd: YAG laser infrared radiation with a pulse width of 6 nm (maximum resolution of 23 *μ*m with a 36 MHz transducer) was transmitted to the sample. The time range photoacoustic signal for each piece of data was measured using a digital oscilloscope. The photoacoustic signal of a pulsed laser is strong enough to increase the amplitude of the ultrasonic signal without the need for a (pre) amplifier. Consequently, the UST is directly connected to the oscilloscope input channel with a predetermined amplitude at the sampling rate. So, the oscilloscope works in the external trigger mode to take simultaneous measurements without delay. The photoacoustic signal starts to be recorded when the output signal from the laser system is sent. So, by using an ultrasonic transducer and an optical fiber to send laser light to the target, the signals from the sample (cholesterol) absorbing the light are collected and sent to the CPU unit and the host computer to be processed.

## 3. Results and Discussion

According to the experimental imaging results, the photoacoustic system has an axial resolution of 46 micrometers. In other words, it was discovered that a delayed photoacoustic signal emitted in water at depths less than 46 microns could not be distinguished using low-frequency signal processing. Increasing the axial resolution of low-frequency acoustics on the reciprocal photoacoustic signal's depth is the current method's objective.

In order to examine this study in greater depth, the effect of various frequencies has been evaluated first. In this regard, frequencies between 100 and 400 Hz are investigated, along with phase and amplitude parameters. The phase spectrum of an open photoacoustic cell for liquid cholesterol is considered to investigate the phase values. The relationship between various frequency and phase values is depicted in Figure 3. It is evident from the figure that the frequency spectrum and the phase spectrum are related. The phase spectrum becomes more compact as frequency increases. The maximum value of the phase spectrum is 58.66 degrees, which occurred at 100 Hz. The lowest value of the phase spectrum is 46.37 degrees, which occurred at a frequency of 400 Hz.

Figure 4 shows the amplitude changes for different frequency values. It is evident from this figure that amplitude and frequency are directly related. The amplitude continues to increase as the frequency increases. The figure indicates that the minimum amplitude value is equal to 1.95 and occurs at 100 Hz, while the maximum amplitude value is equal to 17.67 and occurs at 400 Hz [40].

As seen in Figure 5, the amplitude between the two peaks in the time domain spectrum is diminished due to the time difference between the upper and lower levels of the signal received from the cholesterol-coated wedge. In order to obtain a more precise image of the closely spaced merged peaks, the second derivative is applied to the selected time interval following the application of the algorithm for coherent correlation shear. Notable is the maximum amplitude of 6.36 microseconds, which occurred in 4.09 microseconds, and the minimum amplitude of 0.06 microseconds, which occurred in 8.21 microseconds.

Figure 6 depicts the photoacoustic properties of the 200-micron data using the second derivative. The time difference of the time domain spectra at the speed of sound in water (1.5 mm/microsecond) is multiplied and calculated to determine the two-point distance caused by the laser striking the upper and lower levels. The photoacoustic output spectrum displays the oblique side lobes clearly defined after applying the derived filter [41].

Figure 7 shows the least detectable changes (equal to 46 microns) using the present method. It is evident from the diagram that the two diagrams differ slightly from one another. It is important to note that the maximum amplitude value in this figure corresponds to the blue graph and is equal to 6.05; it occurred in 4.25 microseconds. In addition, the red graph represents the lowest amplitude value, which is 0.22 and occurred in 3.5 microseconds.

Figure 8 depicts the thickness changes of wedges coated with cholesterol oleate. Consequently, this technique, which is based on an orthogonal signal processing algorithm in the frequency domain and the extraction of co-phased and quadratic components by selecting and scanning the time delay created by the shear algorithm, can create clarity in the desired range [42]. It is important to note that this figure's maximum and minimum amplitude values are related to the red graph. Therefore, the maximum value of the amplitude is 5.71, which occurred in 6.26 microseconds, and the minimum value is 0.75, which occurred in 5.5 microseconds.

## 4. Conclusion

For the first time, with a novel approach in this paper, a photoacoustic system for measuring the thickness of cholesterol in blood vessel walls was presented. A low-power, low-frequency, continuous-wave laser was used. In pulse systems, the frequency of controllable pulses is limited, and jitter significantly impacts the final synchronization of the sample and reference signal. The current photoacoustic system has an axial resolution of 46 micrometers. Consequently, it provides significant features for high-resolution medical and industrial systems where high axial resolution is crucial. Most blood vessel disturbances are caused by water, which can be reduced by employing a differential system and complementary wavelengths. Therefore, it is concluded that the combination of fast signal processing units and high repetition pulse lasers increases the resolution to submicron levels for measuring the thickness of cholesterol in veins. With the present method and its expansion and development in the form of a catheter, the primary nuclei of sclerotic plaque can be created and utilized in the early diagnosis and diagnosis of atherosclerosis in high-risk groups and the early prevention of disease progression. Photoacoustic imaging is a nascent method in laboratory research in medical imaging that can be applied to a wide range of physiological and anatomical investigations. Due to nonionizing radiation, this method can eliminate the limitations of diagnostic techniques that rely on ionizing radiation.

## Figures and Tables

**Figure 1:** Photoacoustic effect and production of ultrasound waves [37].

**Figure 2:** The system used in this study [37].

**Figure 3:** Open photoacoustic cell phase spectrum for the cholesterol liquid.

**Figure 4:** The relationship between different values of intensity and frequency.

**Figure 5:** The time range of the photoacoustic system is about time 3.5 and 4.5 *μ*s.

**Figure 6:** Extraction of spectral information after applying the second derivative filter.

**Figure 7:** The lowest value detectable by this method.

**Figure 8:** Two distinct points of the wedge to show the changes.

## Data Availability

The authors confirm that the data supporting the findings of this study are available upon request.
